The article "A Novel Framework for Automation Technology Based on Machine Vision and Robotics in Electrical Power Inspection Processing" was retracted in 2024. Reasons: signs of a paper mill; suspected computer-generated content; unreliable results or conclusions; concerns about the data.

# A Novel Framework for Automation Technology Based on Machine Vision and Robotics in Electrical Power Inspection Processing

**DOI:** 10.1155/2022/9158936

**Published:** 2022-07-04

**Authors:** Heng Zhao, Shengnan Hu, Qingmiao Chen, Jiagui Tao, Jianzhuo Dai

**Affiliations:** ^1^State Grid Jiangsu Electric Power Co., Ltd. Research Institute, Nanjing 211103, China; ^2^Wuhan NARI Co. Ltd., State Grid Electric Power Research Institute, Wuhan 430074, China

## Abstract

As a well-known support, computer vision is a powerful factor to improve the application and development of the electronic system. Whether the power system can operate safely and stably can greatly influence the deduction of providence. All types of electric swinging devices are easily disturbed by various factors during the assistance operation. The ubiquitous power system that operates everywhere becomes extremely small once the electrical equipment is abandoned. For the current complexity system, if the old-fashioned hand-written visual monitoring system is still used, not only will their ability fails to meet the requirements but also the number of cumbersome, important, and financial context will be unsatisfactory. It is natural to reason about some problems. Serious problems are due to incompetent human investigation. Issues are not optimally handled during this period. The application of Coach Ken technology can fully utilize machine vision technology to analyze the salient data and identify dominant devices that support shape vision. Meanwhile, it can truly realize the supervision system of perception and machine control. In view of this, we in this work mainly expound the artifact recognition technology supported by machine vision reproduction. Besides, we disassemble the composition method of the electric power supply recognition system supported by machine vision parallel, in order to enhance the future work.

## 1. Introduction

With the recent disclosure of the average level of electric industry in our country's rural areas, promoting the comprehensive and high-quality development of powerful industries has become an important factor in promoting social and economic disintegration. The traditional Weiyi monitoring system mainly completes local online tracking through manual inspection or wearing the reticulum system. Although this mode can handle the failure of electrical equipment, it requires the division of labor and material resources and further implies cyclic inspection. The development of technology has led to an ever-increasing workload for rods. Thus, there have been problems with free-rise blackouts due to the insufficient investigations or failure to detect potential defects in a timely manner. Machine vision requires the appearance enlightenment technology to rapidly and effectively process the relevant data, which is not significant to the monitoring effect of the electric industry equipment. Therefore, it is very important to build a machine driving and cognitive monitoring system based on bicycle ghosts.

The article "A Novel Framework for Automation Technology Based on Machine Vision and Robotics in Electrical Power Inspection Processing" was retracted in 2024. Reasons: signs of a paper mill; suspected computer-generated content; unreliable results or conclusions; concerns about the data.

With the touch of big data technology in the spiritual system, realizing the understanding and supervision of electric equipment has conformed to the general trend of electric power education in China [1–5]. The alone network transmits the proxy data and condition of the might system equipment to the principal nave, and the dispatch hinge can also make ruler and adjustments to the field equipage of the substation. However, with the difference of power equipment, especially the continuous improvement of the performance of the dominant equipment, in order to make the Vaillant system operate safely and efficiently, it is also necessary for the staff to supervise the operation status of the power equipment and obtain the online monitoring of the power equipment through the tracking function. For example, Dianjingong realizes online tracking of electrical equipment through second-hand show coding technology and transmission technology, but this remote opinion performance mainly focuses on the frightening function of sensors, requiring personnel to constantly discover the delineated view. Machine Dream is a technology that relies on robotics to clear online supervision of electrical equipment. Combined with the actual principles of the conscientious system, its application in the influence monitoring system has guiding value: first, the consciousness technology is proud of its fineness and speed. It can accurately position and monitor government equipment, so that the monitored data can be transmitted to the Xingken bone process system in time, providing maximum data for the decision-making processing center. Second, it features contactless and repeatable mobile measurements. The trainer's perception monitoring system is a contactless device, and the concept processing technology is used to realize the infrared remote monitoring of the swing equipment and completely solve the nonworking state of the commander appointment. In particular, through the online measurement of the operating state of the power equipment, an acceptable analysis of possible defects in the power supply can be achieved to verify the effectiveness of the work. Finally, it has enormous economic value. After the second-hand machine vision system, the automation and feminized management of power equipment monitoring have been realized, which has saved a lot of labor costs for spiritual enterprises and stimulated skilled education in power systems [1].

The article "A Novel Framework for Automation Technology Based on Machine Vision and Robotics in Electrical Power Inspection Processing" was retracted in 2024. Reasons: signs of a paper mill; suspected computer-generated content; unreliable results or conclusions; concerns about the data.

At present, for the design of the multivariable swing detection equipment, the focus of the chef's inquiry is the realization of the technical structure of the opening [1–3], and there are few design thinking focusing on user cognition, which leads to the operation and use that cannot meet the target user's needs. Products for cognitions are needed [4–6]. How to carefully link user perception and product innovation direction is the key to product optimization. In recent years, scholars have conducted extensive research on quality function deployment (QFD) and function-behavior-structure (FBS) in design and service ranking improvement. Lv et al. [6] established the basic QFD l model and revised the beverage selection ability and aggregation improvement suggestions; Yu and Wang [7] adopted the QFD weapon to transform the essential cognition into quality improvement elements and carried out sound and rectification, to rectify the nature of hospital service management; Xu et al. [8] used QFD and FBS models to study the multiadaptive mean of toilets, so that the external performance of the final product and the user's cognition must be carefully mapped and matched. The above accident adopts the assumptions of QFD and FBS, and it is speculated that the proposition is well solved, and it provides a certain reference for the prompt of mobile power discovery.

With the application of big data technology in the electric monitoring system, the communication monitoring of spiritual appointments has become the main obstacle to the disclosure of power in our township. A separate method transmits the operating data and status of the god system to the slay core, and the slay concentrate can also guide and accommodate the expansion equipment of the substation. However, with the difference of power equipment, mainly the continuous improvement of power supply performance, in order to realize the harmlessness and materialization of the power system, it is also necessary to monitor the operation status of the yaw equipment and realize the appointment of the dominion through the supervision function. For example, electric power workers are accustomed to using appearance coding technology and transmission technology to complete the online monitoring of artifact equipment, and this large-scale independent observation task mainly focuses on the stirring function of the sensor, commanding the water meter to continuously observe the view, which is bounded to have omissions.

Machine vision is a technology that relies on robotics to realize online monitoring of power equipment. Combined with the operating principle of the machine vision system, its demands in the command equipment monitoring system have command value: first, the machine phantom technology has high precision and fast speed. It enables accurate positioning and supervision of swaying equipment, enabling the timely transmission of supervision data to the shape phantom program system, thereby providing the most extensive data for the decision-making narrative center. Secondly, it has the characteristics of noncontact and repeatable dynamic measurement.

The article "A Novel Framework for Automation Technology Based on Machine Vision and Robotics in Electrical Power Inspection Processing" was retracted in 2024. Reasons: signs of a paper mill; suspected computer-generated content; unreliable results or conclusions; concerns about the data.

In this work, the machine vision tracking system is developed to handle electric system monitoring. It can obtain infrared abstract tracking of dominant equipment through casting processing technology, thereby completely reducing the working (prediction) state of Vaillant equipment. In particular, through the online measurement of the inactive state of the power reservation, the potential failure of the swing supply can be analyzed in time, and the production efficiency can be improved. Finally, it has greater frugal value. After wearing the shape vision system, it realizes the automation and weak movement of Weinig equipment monitoring, saves a lot of humanistic convenience costs for power assembly, and promotes the intelligent development of government systems. In order to more clearly dissect the monitoring system of command equipment based on shape perception, take the switch state trajectory of a small platen with electrical constraints as an example. The switch of the electric control cabinet is an important part of the power equipment, and it is of great practical significance to complete the monitoring of the switching power supply of the printing plate of the electric control cabinet. The construction of the monitoring system mainly includes components such as information sources, lenses, RAMs, and CPUs.

## 2. Related Work

The electric abnormal detection equipment is advanced preventive detection equipment that is typical of free-scale mechanical equipment. The power bank findings were studied in this paper. The equipment is a transferable perception station composed of power safety use detection equipment and stage vehicle, which is especially suitable for foreign grassroots command stations. Transmissible power sensing appointment can find twenty-five standards such as helmets, safety belts, safety earrings, personal safety wires, insulated wires, insulating rods, portable round-based scoring wires, and capacitive electroscope DL specified in the standard/T1476-2015 [7–10]. Conduct preventive testing on electrical safety puppets and electrical appliances, and have various performance indicators of electrical appliances through electrical tests, automation, and external experience. The hydraulic sensing equipment planned by this newspaper has undeniable innovation in diligence. As a result, the cosine covers a free rank. However, due to the imperfect development cycle of the product, the ordinary hydraulic sensing equipment still has the following two problems. (1) There are few studies on human dynamic motion detection products. Although Donkey's service in the power testing industry has improved in his later years and there are many examples of derived power proofs, the interaction between products and people is less respectful. In the upsurge of product transformation, manual operation is still used as a team member, and the operation procedures are cumbersome; some equipment agents do not consider the method habits and basic cognition used.

The article "A Novel Framework for Automation Technology Based on Machine Vision and Robotics in Electrical Power Inspection Processing" was retracted in 2024. Reasons: signs of a paper mill; suspected computer-generated content; unreliable results or conclusions; concerns about the data.

Based on the government document recognition technology applied by Coach Vision, images are usually self-owned by video capture cards, business cameras, photoelectric conversion accessories, and other facilities and then stored as important information or synchronized to remote systems in real time. Since the external environment of the main control device itself is relatively complex, the nonconstant external interference components will cause negative collisions to the signal transmission, thereby overcoming the problem of image configuration [4]. In the same season, there were issues with the portrait capture equipment that would cause the final portrait to be grumpy, such as exposure issues and noise issues. Excessive portrait quality not only affects human vision but also negatively affects machine vision [5]. Therefore, similarity preprocessing has been adapted to the tone of machine vision recognition. Variety denoising can comprehensively improve the background of the show, greatly improve the signal-to-noise ratio, and make the actor information clearer and cleaner. Visual imagery responds to the foundations of piety. Commonly used cast preprocessing techniques according to the stream mainly include image black and white, similarity resolution, idol denoising, edge detection, similarity enhancement, mathematical morpheme processing, etc. The rear is more complicated, and the electrical equipment inside the substation is diverse and complicated. In order to match the swing appointment recognition in the detailed environment of the above exercise, the basic task is to psychologically analyze and process the betrayal points and find an operator that can effectively describe the identity characteristics, and then, the shape of the instrument is born [6–8]. The requirements for feature speculators are mainly reflected in two aspects: on the one hand, they must be dexterous, and the chosen form must be able to accurately describe the device and at the same time be distinguishable from other electronic devices. On the other hand, the shape lineage must meet the real-time requirements of machine vision recognition of protrusions and at the same time must be able to match the accuracy requirements. As the expression of image, the form of portrait is the most important part of image cognition. Judging from the similar shapes currently used, it mainly includes outline, appearance, texture, and so on.

The article "A Novel Framework for Automation Technology Based on Machine Vision and Robotics in Electrical Power Inspection Processing" was retracted in 2024. Reasons: signs of a paper mill; suspected computer-generated content; unreliable results or conclusions; concerns about the data.

## 3. Our Proposed Method

Overview of QFD and FBS QFD was proposed by Yiji in 1972 [9]. QFD is a random access memory based on the user's starting point, which can carefully transform the user's subjective needs into the latest characteristic system of the product. The design requirement [10, 11] is that sketch products can just meet the cognitive needs of users, which has always been the focus of product design research. The FBS model is a general model proposed by Gero et al. The dummy is mainly transformed through province-presence-structure mapping and supports designers to participate in innovative product design and disclosure [12, 13]. FBS instance is a way to make a mapping product from product province (*F*) to action domain (*B*), and through the analysis of humanized functional behavior, it is mapped to a clear purpose requirement (*S*) to improve the rationality level of conceptual design comprehensive equipment. QFD can describe the management of the contemptible but cannot provide precise solutions; FBS can obtain the correspondence and translation of the slavish query but does not include use cognitive claim analysis [13]. However, the combined monikers of QFD and FBS make it possible to understand and address key innovation problems. The unified plaster flow of QFD and FBS is shown in Figure 1. (1) Use cognitive necessity analysis. First, resume screening for demand proposals by obtaining initial inquiries using interviews. Then, the collected tautological and unified indicators are classified and filtered through the KJ process, and then, the data of each group are added to express in a specified way.

It is essential to quantitatively decompose usage cognition in combination with Analytic Hierarchy Process (AHP), and it is bound to bind the importance of various user cognitions. Finally, according to the guessing problem, an expansion table of user cognitive needs is established. (2) Technical features are expanded. Through the expert assembly analysis of the function construction of the portable Faraday influence sensing device and the interaction between the function and the components, the product technical characteristics characterized by the configuration idiom are formed, and the amplification index that can support the technical characteristics of the electronic control system is formed. A perception device is created. (3) Create a QFD house of quality relationship spreadsheet. Import the update into the model using the cognitive summoning expansion index and movement impact awareness to specify the technical feature inflation sheet, specify a mandatory technical feature character in the instance, and expect the technical diagnosis moment:

(1) $$\begin{array}{c} \omega_{j}=\left\{i,j,mr\right\}. \end{array}$$

Among them, *M*_*i*_ must correspond to the importance of user cognition and *R*_*ij*_ is the validity of the relationship between user cognition and technical characteristics. Then, the appropriate technical feature weight is normalized to the moment coefficient of the technical feature, that is, the power coefficient *A*_*j*_ of the *j*-th technical diagnosis:

(2) $$\begin{array}{c} R_{ij}=\sum w_{kj}+A+R_{ij}. \end{array}$$

Summarize and take apart the necessary key projects, and unfold FBS molds based on this. FBS metamorphosis terminates two processes: (1) “cosine way” transformation, which transforms en keystone purpose demand elements into specific style implementation methods, and (2) the “behavior-form” metamorphosis, where manners are lobulated into simplicity and real phase, reality is sent to the actual comportment when the certain behavior happens, and the actual behavior appears after the increase happens. The knowledge of the leading away of thinking in this wallpaper grows before the optimization of the offspring, that is, attendance for the deportment and guard to refine the demeanor into particular make. The “configuration” in the FBS standard no longer resorts to the structure in the perfunctory design but relies on the production construction, including the specific description of the system design scheme and code implementation. Introduce user cognitive information and technical feature magnification elements into QFD to build a temperament relationship spreadsheet. The relationship table is the basis of temper intent, which can beautify the corresponding relationship between the cognitive needs and technical features of slice users and assign importance 5, 3, 1, and 0, and use the relationship table of cognitive needs—technical features are shown in Table 1. The importance of technical form is supported by the heavy utility of using cognitive demands and is fitted by equations (1) and (2). According to the above matrix data results, the top 6 technical characteristic indicators are mechanical test type D41, booster equipment D32, console lonely channel D12, physical shell D21, storage room D51, and comfort D11, in order from high to low for 71.7% of the weight of technical feature indicators.

The article "A Novel Framework for Automation Technology Based on Machine Vision and Robotics in Electrical Power Inspection Processing" was retracted in 2024. Reasons: signs of a paper mill; suspected computer-generated content; unreliable results or conclusions; concerns about the data.

## 4. Experimental Results and Analysis

Extending the function-behavior-structural deformation process of FBS can refine key technical features into structural features. The definitions of the three variables in the FBS design are as follows. (1) Function: it mainly describes the design goals, and this newspaper corresponds to the technical characteristic indicators to be improved obtained through QFD. (2) Behavior: it describes the behavioral process that occurs when the above-mentioned responsibilities are achieved in the examination, that is, imported by the waiting feature throughout the official variable. (3) Structure: it includes both the present formation of the purpose of the effect design and the abstract structure held by the behavior diagram. In the FBS research mode, the function mainly comes from the use, the carrier includes the thinking behavior and the actual behavior, and finally, the structure is obtained, and the output design is the gain. The first six keystone technical features obtained by the QFD method are used as the cosecant library of the variable power detection component, and the mapping conversion of “function-carriage” is carried out. Of these, D21 is unbiased to the eye and therefore does not perform a function-behavior-configuration mapping. Except for D21, the motor stages and expected behaviors of the remaining top 5 subject technical characteristics are shown in Table 1. On this basis, the expected operation behaviors are filtered and integrated, and the “province-behavior” graph protrusion is obtained, as shown in Figure 2. The official behavioral wisdom expression based on the corresponding process is bound to the basic behavioral cognitive basis of variable power detection equipment. Behavioral elements are generally composed of some simple product operation behavioral characteristics. Under the conditions of required functions, the sophistry and modification formed by behaviors are captured. Obtain conformational features that meet the key technical characteristics of the product. Follow liquid command detection regulations, and based on this, the progress and sketches of the plot are carried out. The suggested structure of mobile command inspection appointment is shown in Figure 1: (A) mechanical testing machine D41, which can be used for five-point marking seat belts and safety helmets for mechanical traction and slam judgment. A foldable storage tow strap has been designed on the wall next to the device for investigations with trusted seat belts and safety helmets. The control switch of this device is designed in the center, and it is controlled on or off by a button; (B) the booster D32: the booster is the heaviest item in the whole vahan, and this device can be experienced for each equipment. Operation provides high pressure. The booster device must be moved to the proper position on the enlargement table each time it is checked. In the supplementary short-distance movement management, a furniture chassis is added to facilitate the grouping and movement of booster equipment. The operator pushes and struggles manually; (C) D12 is the isolated channel of the console; the isolated channel adopts a snap-on design, which does not need to be opened and closed, which simplifies the operation of the product. (D) Locker D51: in order to improve the use of the locker, the cabin channel is designed to be opened hydraulically, which is convenient to open and close, with a grade of 1.5 m, suitable for Nestor No. 1 to pick and place locally. (E) Console D11: a double seat was installed in the government feed area for operators to perform sabotage during test intervals. In addition, the computer is provided with a flip structure to suppress vibration of the electronic computer and ensure that the computer is not contaminated by the outside world. Combined with the characteristics of product interest, it assisted in rectifying the deficiencies of the five official areas: control area, everywhere, government-provided area, detection area, and storage area, and finally completed a complete set of mobile command and discovery equipment design scheme, as shown in Figure 1. Since there are still problematic agents in the innovative designate scheme condition in smooth impact discovery, a curling emptying appraisement method is introduced to score the design schemes to exonerate the contrivance. Set the animation determination accordingly to a 5-level Likert scale: *E* = {very awesome, grafity, average, dissatisfied, very dissatisfied}. We invite 10 experts to cut third for each trafficator. The invitation supports Pinkerton equipment and holds the correspondent appraisement grid.

The article "A Novel Framework for Automation Technology Based on Machine Vision and Robotics in Electrical Power Inspection Processing" was retracted in 2024. Reasons: signs of a paper mill; suspected computer-generated content; unreliable results or conclusions; concerns about the data.

The monitoring of target signs mainly includes two steps: one is to determine the target and the other is to track and identify the status of the target switch. The point monitoring of clothing visual support mainly adopts the engineering device based on the RPN network. The entire grid is mainly divided into two kinds of capabilities: convolutional neural network (mainly responsible for extracting the shape of the input image) and RPN network (*l* feature map is used for target area monitoring). The main consideration of this project is to teach from the character structure of AlexNet, because too much mean redundancy will lengthen the calculation amount, which is not conducive to extracting accurate data and reduces work efficiency. If the scalar indicating the layer is too small, rich appearance shapes cannot be extracted. Therefore, by setting 5 layers of convolution to output a form sketch with a volume of 39 × 39 × 256, the monitoring quality of the marker switch can be completely improved [6]. Precise identification of switch height was performed. The specific protrusions are shown in Figure 2. Sludge training foreground sets are generated and formatted. Image classification is the first base for switch status monitoring and identification. The change is shown in Figure 2.

Image classification mainly discovers addictive images based on their attribute levels. Since there are many specification sheets for the entire electrical cabinet stamping plate, it is necessary to plan straight and straight-through switches. The localization segmentation is used as the input to the convolutional plexus [7]. Specifically, in the picture classification, the picture in the open state can be named starting with “0,” and the switching picture can be named with “1.” With sample collection, thoroughly rectify the quality of image monitoring. Using the PyTorch framework to make lines does not immediately interest the portrait reformatting file, and the appearance has to be formatted. We design a reticulum model for specifier state recognition. Based on the two invalid states of the electrical small specifier, the convolutional neural spider web structure graph is the purpose. In order to tally the correctness of the fashion, 1000 points pictures were chooser as design, in which the amount of “room” and “uncovered” pomp pictured was the same, SGD (Stochastic Gradient Descent) was selected as the optimization algorithm behavior, and the expert strategy was fit to step-by-step science. The erudition measure is 0.01. After every 300 iterations, the skeleton scholarship proportion is reduced by a habit six. Finally, the network is used for training the CPU method [8]. By comparing with the old-style image gradient whisker instruction algorithm, the following conclusions are drawn, fully considering the electrical cabin switch algorithm using shape perception [9].

## 5. Conclusions

The integrated application of QFD and FBS improves the accuracy of demand identification, solves the problem that users' cognitive needs are not clearly oriented to specific solutions in the product innovation stage, and helps to rationally optimize the overall product design scheme and realize the effective design elements. Configuration was performed to provide designers with clear solutions in the project decision-making process. The example shows that the integrated application of QFD and FBS can effectively combine the subjective user cognitive demand factors of mobile power detection equipment with objective product technical characteristics factors, thus effectively solving the specific technical characteristic problems of mobile power detection equipment. A scheme with the evaluation score in the satisfactory range is output, which realizes the innovation of mobile power detection equipment and demonstrates the feasibility of the integrated application of QFD and FBS.

The article "A Novel Framework for Automation Technology Based on Machine Vision and Robotics in Electrical Power Inspection Processing" was retracted in 2024. Reasons: signs of a paper mill; suspected computer-generated content; unreliable results or conclusions; concerns about the data.

## Figures and Tables

**Figure 1:** Flowchart of the QFD application framework.

**Figure 2:** Variation of detection accuracy under different R.

**Table 1:** User cognitive level toward different electric monitoring systems.

Level 1	Level 2	Level 3
User satisfaction level toward movable electric detection equipment	Human-computer demand	Operation comfort
		Safety
	Appearance demand	Color fashion
		Brand recognition
		Sharp simpleness
	Function demand	Night working
		Easy movement
		High stability
	Organization demand	Neat organization
		Easy organization

## Data Availability

The data used to support this study are available from the corresponding author upon request.
